This article has been retracted.

# Design of Teaching Quality Analysis and Management System for PE Courses Based on Data-Mining Algorithm

**DOI:** 10.1155/2022/6830375

**Published:** 2022-05-31

**Authors:** Sen Li, Yanrui Luo

**Affiliations:** School of Physical Education and Health, Shanghai Lixin University of Accounting and Finance, Shanghai 201620, China

## Abstract

Advances in network technology have led to extensive information technology construction work in all walks of life; universities, as a key component of national development, cannot be overlooked in this regard. In today's universities, the Web-based integrated academic management information system is widely used, promoting higher education management system innovation and improving the management level of education departments and teaching management. The traditional management mode is incapable of locating “knowledge” in the mountains of student transcripts, and the original management mode must be improved. In business, finance, insurance, marketing, and other fields, digital exploration technology is widely used. This article describes the design approach for a data mining-based analysis and management system for PE course teaching quality, as well as the application of information technology and data mining technology in PE by combining actual PE teaching in schools, with the goal of realizing a data mining-based PE performance management system to serve PE teaching in schools and improve PE teaching quality. The results show that the time required to find frequent itemsets using a traditional algorithm running on a single machine, as well as the time required to scan the database several times for frequent itemset search in a distributed cluster of 20 computing nodes, is significantly longer than that required by the data mining algorithm. As a result, the proposed sports performance management system is functional, simple, and scalable, with each functional module operating independently and cooperatively, reflecting the concept of “high cohesion and low coupling.”

## 1. Introduction

Along with the expansion of college operations, the number of students is increasing year by year, and the teaching of physical education, which is an important part of school education, has sparked a wave of pedagogical reform [1]. Classroom teaching is the primary means of achieving educational goals in schools, and its effectiveness has a direct impact on the learning quality of students [2]. Colleges use improving higher education quality and cultivating special talents as the purpose of school operation in order to respond to the national call and achieve the state's higher education development goals [3]. The original grade data analysis method, on the other hand, is unable to thoroughly analyse and capture information useful for teaching and learning from large amounts of grade data, resulting in inefficient use of teaching information resources. This has resulted in grade management based primarily on simple statistical analysis, such as processing student identity. Data mining [4, 5] is a vital information processing technique [6, 7] that has been widely adopted in a variety of industries around the world, generating significant economic and social value.

The service that universities provide to students as a “service-oriented enterprise” is “education.” We can only “produce” a high-quality product—graduates—and establish a brand name in the education market by continuously and effectively improving education quality [8]. Knowledge and rules in the knowledge base are created by experts or programmers using external input in traditional decision support systems [9]. Data mining is an automatic process of acquiring knowledge from within a system with the goal of discovering undiscovered knowledge in a large amount of data [10]. Online query and analysis can be used to process information that is clearly understood by decision-makers [11]. It is beneficial to motivate teachers, improve teaching quality, and strengthen faculty construction and scientific management by establishing a good teaching quality evaluation mechanism [12].

Many schools now conduct physical activity and achievement tests for their students [13]. The majority of these post-test scores, however, are only saved as data or files in school computers, and these students are unaware of their physical condition despite having completed the relevant physical fitness tests [14]. Analysing and processing these massive amounts of data using traditional data analysis and data query validation methods are not only computationally intensive but also completely reliant on pre-assumed and estimated data relationships. In data, there is a growing demand for tacit knowledge [15]. The use of parallel computing and data-mining arithmetic can help to solve this problem to a large extent, because parallel computing can provide the computational power required to process large amounts of data, and clusters can scale up the computational power as the data grows. In response to the problems and current state of PE in universities, relevant information is compiled, and modern data mining techniques are fully employed to automate the processing and analysis of large amounts of sports data in order to assist students. Professors and consultants analyse statistical data. In this paper, technology for digital exploration is introduced into the performance analysis of the university teaching system, with the goal of identifying factors affecting students' performance and specifically improving teaching quality. The innovative points of this paper are as follows:

1. Using data mining techniques to uncover possible hidden relevant factors that affect teachers' teaching level, provide specific indications for improving teaching level, and apply them to teaching practice.
2. Research and analysis of existing student data information using association rule extraction technology, and statistical analysis of some factors affecting teaching quality in schools using scientific methods, so as to evaluate teaching quality and student learning quality.
3. The purpose of the analysis and management system of PE curriculum with quality according to data mining algorithm is to enhance the productivity and accuracy of PE teachers in schools, free them from tedious and boring work, and then improve their management-level teaching quality.

The first part of this paper introduces the background and significance of the study, and then introduces the main work of this paper. The second part introduces the work related to the teaching quality analysis and management system of PE courses, data-mining arithmetic. In the third part, the system functional module design and the logical system design of the physical education database are explained so that the readers of this thesis can have a more comprehensive understanding of the design idea of the physical education curriculum teaching quality analysis and administration system based on the data mining algorithm. The fourth part is the core of the thesis, which describes the usage of data mining algorithm in the quality control system of physical education from two aspects: data point set compression and discard analysis and large-scale data set clustering process analysis. The last part of the thesis is the summary of the full work.

## 2. Related Work

### 2.1. Quality Analysis and Management System of PE Course Teaching

To enhance the cultural qualification of all the people, China's higher education has made rapid progress, with major breakthroughs in system reform, successive expansion of various colleges and universities, and leapfrog development in the scale of college operation. However, it is impossible to implement the national education policy, let alone to implement quality education, if the physical health training of young people is neglected. Therefore, classroom teaching quality monitoring has great significance as an essential component of the university's education quality supervision mechanism, and the study and improvement of the teacher classroom teaching quality evaluation system is one of the hot spots and priorities of the current higher education evaluation of quality management.

From the perspective of effectiveness, Cao defined teaching quality evaluation as the evaluation process, which is essentially the process of determining the extent to which curricula and learning programmes actually achieve educational goals [16]. Cui and Yoon proposed a decision tree data extraction method that combines this algorithm with the SLIQ algorithm and applies it to a database of student grades to analyse various data and build a decision tree model through analysis [17]. Parmezan et al. proposed a teacher teaching quality assessment questionnaire that includes nine dimensions such as teaching quality, value of learning, enthusiasm for teaching, teaching organization and clarity, group interaction, interpersonal harmony, breadth of knowledge, examinations and test scores, homework, and other reading materials [18]. Zhang et al. conducted an in-depth study on mining techniques and proposed the ID3 algorithm to manage the university faculty-related data was extracted and analysed to discover correlations between various course environments with a view to providing data university decision reference [19]. Yin discussed the application of distortion-resistant algorithms in mining association rules. This algorithmic technique significantly reduces the number of database scans by a factor of even less than two. The algorithm with the shortest scanning time is the use of sampling to collect relevant data [20].

Teaching quality analysis is an important tool for evaluating teaching and learning. Data-mining arithmetic is used to analyse data generated from examination processes and teaching sessions at multiple levels and perspectives. Utilizing the analysis results to assist teaching decisions is an inevitable requirement for assuring teaching excellence and enhancing the quality as well as the overall competence of students and teachers.

### 2.2. Data-Mining Arithmetic

Given the current rapid development of higher education, self-monitoring of school teaching quality has become an important guarantee for scientific administration, and the development and implementation of teaching quality evaluation systems has become an important tool for implementing teaching control. Currently, digital exploration technology is widely used in telecommunications, commerce, banking, and enterprise production and marketing, but it has a limited use in education. As a result, this research focuses on the performance analysis characteristics of PE courses and integrates them with practical work to propose a data mining-based algorithm for identifying the keys that have the greatest impact on students and enhancing their learning experience. Dan and Li classify the original data set for large-scale data sets, analyse the OS virtual memory implementation mechanism, and improve the original FP-GROWTH algorithm in terms of spatial and temporal locality to make it a mining algorithm with perceptual input and output [21]. Gong and Lin proposed a multivariate strategy, which combines previous mining and discovery techniques and applies them to the qualification database to help universities make better decisions. To assist teachers in making teaching decisions, the results of each subject are computed, as well as a performance analysis report and related analysis table [22]. The hardware and software infrastructures for distributed association rule mining algorithms were investigated by Atta-ur-Rahman and DaSh. They looked at distributed data mining algorithms, parallel mining algorithms, and distributed parallel databases [23]. Li et al. discussed the Apriori association rule algorithm and the well-known decision tree ID3 algorithm, as well as their application scope [24]. Huang used a similar algorithm, Random-kmeans [25], to sample the original data set statistically and pool the smaller data set after sampling. The relationships and trends that are hidden in large amounts of data are beyond the ability of even the experts who manage these data to discover, and this information is potentially and critically important for decision-making, which is what data mining aims to solve.

## 3. Design Ideas of Teaching Quality Analysis and Management System of PE Courses Based on Data-Mining Arithmetic

### 3.1. System Functional Module Design

An important task of the generic system design phase is to determine how the system will accomplish the intended functionality using a more abstract and generic approach [26]. Thus, the overall design phase has three main subphases, starting with the test type management module, followed by the test project management module, and finally the result management module. Data mining is the complete process of extracting previously unknown, valid, and useful information from a database through data mining tools and using this information for decision-making or knowledge enrichment. The system functional module diagram is shown in Figure 1.

First, the test type management module completes data preprocessing [27] and management of sports event types, including adding, modifying, deleting, and configuring the weights of event types. Data preprocessing is mainly done by cleaning, integrating, selecting, transforming, and conceptually layering data attributes to form tuples from the data training set. The information entropy of sample classification is as follows:

(1) $$\begin{array}{c} I\left(x_{1},x_{2},\ldots ,x_{n}\right)=-\sum_{i=1}^{n}p_{i}\log_{2}p_{i}. \end{array}$$

The construction of the teaching quality evaluation system includes two aspects: the determination of indicators and the determination of weights. Indicators are specific, measurable operational and behavioural goals of a particular aspect; that is, they do not reflect the complete goal, but only one aspect of the goal. Simultaneous comparative analysis of factor data of different dimensions requires their standardization. The value of *i* factor *j* in all samples is as follows:

(2) $$\begin{array}{c} Z_{i,j}=\frac{X_{i,j}-\mu_{j}}{\sigma_{j}}, \end{array}$$

where *μ*_*j*_ is the mean value of the *i* th factor and *σ*_*j*_ is the standard deviation of the *j* th factor.

The business problems to be mined are identified by a detailed understanding of the raw data to be extracted and the business problems to be applied in practice before starting data mining. In data mining, determining the purpose of mining is crucial. Mining produces unpredictable results, but the problem to be mined must be predictable, and mining blindness must be minimized. It is necessary to determine whether the test type contains test elements. It is impossible to remove something that already exists. Otherwise, the deletion procedure is carried out.  Figure 2 depicts the programme flow for performing this function.

Secondly, the evidence project management module completes the operations of adding, modifying, deleting, and setting weights of sports evidence items. Due to the large amount of data, among these data, the required data suitable for this data mining are selected to establish a data mining library [28]. It generally includes data selection, selection of relevant data, noise, data purification and elimination, inference of missing data, conversion of discrete-valued data to continuous-valued data, grouping, and classification of data values. Each itemset needs to carry a decision attribute *d*, and when performing a join to produce a candidate *k*+1 itemset, two frequent *k* itemsets that can undergo the join operation must satisfy

(3) $$\begin{array}{c} \left(l_{a},l_{h}\right)\in \left\{\left(l_{1},l_{2}\right)|\text{diff}\left(l_{1},l_{2}\right)=1,d_{1}=d_{2}\right\}. \end{array}$$

As a result, the test management module enables the administration and maintenance of classroom quality assessment programmes, as well as the adjustment of the number of test questions or test content as needed. An independent internal hierarchy to describe the functions or characteristics of the system is created based on the requirements of the questions, and a judgement matrix of higher-level elements is created by comparing the relative importance of factors or objectives, criteria, and plans. To get a sequence of relative importance of relevant elements to higher level elements, a recursive hierarchy is built. Confidence thresholds must be set in order to extract rules from a set of frequent items and calculate the confidence level of the bar rule when extracting sports databases using the active search mining algorithm.

(4) $$\begin{array}{c} \text{Confidence}=\frac{\text{support}}{\left|\text{matched}\right|}. \end{array}$$

Finally, the score management module completes the operations of adding, modifying, deleting, querying, exporting, and grading system conversion of students' sports test scores. The incomplete, noisy, and random data are sorted out, and the unwanted data are cleaned. Suppose *S* is the set of *s* data specimens, and the expected amount of information required to classify a given sample assuming that the class label attribute has a distinct value

(5) $$\begin{array}{c} I\left(s_{1},s_{2},\ldots s_{m}\right)=-\sum_{i=1}^{m}\log^{2}\frac{s_{i}}{s}. \end{array}$$

Then, according to the data mining objectives and data characteristics, appropriate analysis models are selected for the data-mining arithmetic and the data are transformed. The module can classify courses. Different assessment items can be set for each course type. For courses that do not require assessment, you can also set up multiteacher classes to allow for more specific assessment of students. Relevant factors are broken down into levels based on their attributes from top to bottom, with each factor at the same level being subordinate to, or having an influence on, the higher level factor, while dominating the lower level or being influenced by the lower level factor. Then, using a prototype system, developers brainstorm with users to iteratively modify and expand the prototype until the final system is formed.

### 3.2. PE Database Logic Design

The database logical design determines the overall performance of the database and its applications, tuning location [29]. If the database logic is poorly designed, all tuning methods will have limited effect on improving the database performance. The flow of data mining is shown in Figure 3.

First, the conceptual structure is transformed into the corresponding data model, such as relational model, network model, and hierarchical model. The data are cleaned, synthesized and filtered from data sources, and then entered into the database for data mining, pattern evaluation, and knowledge representation. According to the level of abstraction of datum in the proposed rule, association rules can be classified into single-level correlations and multiple-level correlations. KL scatter, also known as relative entropy, is used in the field of statistics to calculate the degree of agreement of two probability distributions, and in the area of machine knowledge to measure the closeness of two functions, and is calculated as follows:

(6) $$\begin{array}{c} KL\left(p\left\|\right)q\right)=\sum p\left(x\right)\log\frac{p\left(x\right)}{q\left(x\right)}. \end{array}$$

Single-level association rules do not consider the hierarchical nature of the actual data attributes, but simply describe the attributes of the data [30]. Metadata is the core of the data warehouse and is used to store data models, define data structures, transformation planning, data warehouse structure, and control information. The management part includes data security, archiving, backup, maintenance, and recovery. The index interval [*a*, *b*] of the soft constraint is given based on empirical data and detects whether there exists a solution within the initial solution set *T* that meets the requirements of the soft constraint. If it exists, it is marked as a feasible solution; otherwise, the parameter range of the constrained indicator interval is adjusted until a feasible solution exists; assuming that *B* is a diagonal matrix, the above formula can be transformed into the following form.

(7) $$\begin{array}{c} e\left(y,z\right)={\left[\sum_{j=1}^{p}b_{ij}{\left|y_{j}-z_{j}\right|}^{s}\right]}^{\left(1/2\right)}, \end{array}$$

where *b*_*ij*_ represents the *i*, *j* data attribute in the database.

In this step, data will be extracted and integrated from the operational environment, semantic ambiguities will be resolved, dirty data will be removed, etc. The process of summing data and calculating data averages are both statistical methods, and the results of these calculations are represented by certain graphs, such as histograms and pie charts. The absolute value function of the factor coefficients in the regression equation is added to the model as a penalty term to make some regression coefficients smaller. By regression, the coefficients of factors whose absolute values are not sufficient to explain the dependent variable can be changed directly to 0. The expression of the LASSO method can be written as follows:

(8) $$\begin{array}{c} \bar{\beta }=\arg\;\min\left\{{\left\|Y-X\beta \right\|}^{2}+\lambda \sum_{j=1}^{p}\left|\beta_{j}\right|\right\}. \end{array}$$

Next, these data models are converted into data models that can be supported by the corresponding database management system. First, all frequent itemsets in the data set are found, and the itemsets that satisfy the minimum support threshold are called frequent itemsets, and then, association rules are generated from these frequent itemsets, mainly by extracting frequent itemsets from all the generated high confidence levels. As a large amount of detailed and descriptive data is stored in the data warehouse, the data set is relatively large and requires a large number of join operations between relational tables to respond to the user's analysis request, increasing the response time user. But the data are stored only once, saving space compared to MOLAP, and analysis can get more detailed data; that is, the granularity of analysis can be relatively fine. So, the branching of attributes is carried out cyclically, and the information gain is the entropy compression expected after knowing the value of the attributes, which is given by the formula:

(9) $$\begin{array}{c} \text{Gain}\left(A\right)=I\left(s_{1},s_{2},\ldots s_{m}\right)-E\left(A\right). \end{array}$$

The database is logically divided into several disconnected blocks, each of which is considered individually and for which all frequency sets are generated. The generated frequency sets are then combined to generate all possible frequency sets, and finally, the support of these element sets is calculated. It is possible to distinguish the similarity of tedious repetitive data in the database, and feature vectors can describe the relevant data with high similarity in the database. The variation parameters of the different features of the data attributes can be calculated using the following formula:

(10) $$\begin{array}{c} e\left(y,z\right)={\left[\sum_{j=1}^{p}{\left|y_{j}-z_{j}\right|}^{s}\right]}^{\left(1/s\right)}. \end{array}$$

Finally, the association rules are verified and the transformed model is optimized. If the extracted rules meet the evaluation mechanism's requirements, the knowledge is sent to the evaluation system and stored in the knowledge base. The knowledge is also stored in the knowledge base if the extracted rules do not meet the evaluation system's requirements. The indexing strategy, data storage location, and storage allocation operation are all determined. Data modelling is needed after determining the data warehouse information to be searched to determine the process of extracting, cleaning, and transforming data from data sources to data warehouse, analysing and dividing dimensions, and determining the physical data storage structure. The primary goal of grade data processing in the academic affairs system is to unify and disambiguate data types. Data decomposition reads data from segmented blocks into memory for processing and then merges all processing results, overcoming the memory bottleneck and improving data set extraction efficiency.

## 4. Analysis of Data-Mining Arithmetic in PE Teaching Quality Analysis and Management System

### 4.1. Data Point Set Compression and Discard Analysis

When the data-mining arithmetic performs in-memory clustering, the data point set is clustered in general and the resulting clusters are marked as the main clusters, and then, the data set in the main clusters is discarded and compressed for deletion. The main memory space reads the data to be clustered again and continues clustering until all clustering work is completed. By setting the maximum available size of the programme, it is shown that this data-mining arithmetic can extract association rules for large data sets in a small memory space. A comparison of the system CPU and GC activity is shown in Figure 4.

First, the discarding process is completed in two steps, which are called primary discarding and secondary discarding. The IP of the data node is obtained from the configuration file, so each node must be a static IP address. The specific configuration table of IP of this system is shown in Table 1.

The main idea of these two discard processes is to move the points that do not change the cluster attributes out of the main storage and store them in the discarded data set. The points in the marker set are not involved in this process and always guide the mining process. Information entropy, called entropy in information theory, is used to measure the average value of the transmitted information. Here, since the process of generating frequent itemsets from candidate itemsets must pass through the database, the most critical part of this process is how to generate the minimum number of candidate itemsets correctly. Therefore, for processing, users classify the data according to their needs and then extract the different parts, thus increasing the extraction speed. The statistical experiment time also does not include the time to write the discovered itemsets to disk in order to accurately count the running time of each algorithm. The support levels are set to 5 and 10, and each algorithm is executed 5 times at each support level, and the average of the statistical record execution time is shown in Figure 5.

Secondly, the main idea of the compression process is to replace high-density regions during the pooling process to clean up the main storage space. It divides the recommendation process into two parts: offline and online. The offline part constructs a cluster using the similarity between users and uses the average rating value of the users in the group as the centre of the group. The set of data points within this region has the same category affiliation and the categories change as a whole. The breast cancer data set was preprocessed, and files of different sizes were obtained by backup. Each file size is approximately 150 million and contains 2 million transaction records. Three *D*_1_ to *D*_3_ data sets were defined, and their specific configurations are described in Table 2.

While the traditional algorithm for finding frequent itemsets using a single machine running a distributed cluster of 20 compute nodes requires multiple scans of the database, the data-mining arithmetic can complete the task of finding frequent itemsets with little time consumption. It only needs to scan the transactional database twice, and does not generate a large number of temporary intermediate key-value pairs, and takes advantage of parallelization very efficiently.

Thus, it can be considered as a whole and can keep its grouping information and have sufficient statistical information. According to the rules defined by the data definition component, the data from the data source are extracted into the data warehouse, cleansing, and transformation; integration work is done; the data are loaded into the data warehouse; the data warehouse data are periodically cleansed; inconsistencies between data are eliminated data storage and source databases; and invalid data are eliminated. A basic principle is that when a transaction does not contain a large set of length *k*, it should not contain a large set of length *k*+1. The information transferred at the source consists of a limited number of mutually exclusive joint complete events, all of which occur with a certain probability. The effect of the size of the data set on the clustering algorithm is tested by varying the size of the data set and fixing the size of the storage space. The results are shown in Figure 6.

Finally, when semisupervised clustering is performed for the data points, labels, SS, and OUTS in the main memory, the data points contained in them are not involved in the compression and discard, thus allowing the set to guide the mining in the main memory all the time. If the description is a model of linking relationships between pages, the logical description can be in the form of a matrix. When mining with aggregate data not only does the mining time increase accordingly, the useful rules are drowned in a sea of rules that are not of interest to the user, but there may be rules that cannot be mined due to the “dilution” of the overall data. Each element of the matrix indicates whether the node represented by the matrix row label to the node represented by the matrix column label is related, which is the hyperlink between the pages in the domain. If the consistency index test passes, the consistency design of the judgement matrix is reasonable, and the corresponding weights reflected by the feature vector are also relatively reasonable.

### 4.2. Analysis of Clustering Process of Large-Scale Data Sets

For a certain scale of transaction database, which contains a particularly large number of candidate itemsets, a transaction can also contain many candidate itemsets, so the number of candidate itemsets will be the main factor limiting the performance of the algorithm. Therefore, it is necessary to choose a large-scale data set clustering process to abstractly describe the various network linkage relationships in reality. At the same time, it is necessary to find a suitable data structure in a high-level language to store the mathematical model in a structured way in the computer, which is easy to analyse and process in the high-level language. To compare the performance of DISK-MINE, DRBFP-MINE, and data mining test algorithms on large-scale data sets, experiments were conducted using a combination of records generated from 2000 different items, and the comparison results are shown in Figure 7.

First, data points from the data set are sequentially read (or otherwise read) into a finite memory called a pipeline until the pipeline's space is filled. The distance between data points is calculated, the data's neighbourhood is determined, the sample's centroid is determined based on the density of the neighbourhood, and the data's global centroid is determined for sampled data. Based on the sample centroids' data, the criterion for selecting the attribute is the information entropy. The information entropy value is calculated based on the data, and then, the sizes of each information entropy are compared, with the largest information entropy being chosen as the selection criterion. The element's information entropy is calculated, and it serves as the decision tree's root node. While all variants of the one-level correlation rule ignore the fact that practical data are multilevel, the multilevel character of the data has been adequately taken into account in the multilevel correlation rule.

The data points in the pipeline are then subjected to semisupervised clustering on finite primary storage until convergence. The entropy value of the system is minimized after using this property to divide the example set into subsets, and the average path from the nonleaf nodes to each descendant leaf node is expected to be the shortest, resulting in a small decision tree. The proposed data to be handled will be related to multiple dimensions using multidimensional correlation rules. In addition, the set of points removed from the main storage goes through a triad after each stage of the discard and compression process, preserving the data point information and grouping information. Density validation and sampling centroids can be done in order, but this takes a long time with large sample sizes and long sampling times, and the sample validation centroids are useless. As a result, it is necessary to consider various influencing factors and compensate each factor appropriately, integrate factors with similar influence, and consider the distribution width and representativeness of factors appropriately during the actual evaluation operation. The comparative analysis of clustering time with positive and negative constraints is shown in Figure 8 to study the influence of the amount of information of equivalent partial constraints on the quality of clustering results and clustering efficiency.

Finally, the data points in the pipeline are compressed and discarded. The data point sets that satisfy the compression conditions are replaced and the corresponding data points are removed from the main memory. The higher the entropy of a training sample set in terms of target classification, the messier and messier it is; the lower the entropy of a training sample set in terms of target classification, the clearer and more ordered it is. The correctness of the algorithm is guaranteed by all possible frequencies established at least in the given block. The online part first calculates the similarity between the target user and the centre of the cluster, then divides the target user into the most similar clusters, and finally finds the nearest neighbours of the target user in the cluster, and then performs item recommendation. In this process, the data points in the algorithm design set can change the attributes of the clusters and also allow new clusters that were not originally in the original set to appear, avoiding wrong labels in the initial set and making the algorithm somewhat fault-tolerant.

## 5. Conclusions

PE to serve the daily physical education in school is an integral step in today's information age. Student evaluation is the system that makes up the most of the teaching quality monitoring system at universities and plays the most important role. The common practise is to use information technology and network technology to assess and predict teaching quality. The ability to apply complex statistical methods and calculations to these data and the rapid access to big data by data mining provide exciting reasons for the rapid development of data mining. Data mining techniques in teaching management, particularly in teaching quality evaluation systems, will provide some data support for university administrators, allowing them to improve teaching quality and make more effective decisions. Using computers to evaluate teaching quality can simplify and improve management. In this paper, we propose a data-mining arithmetic-based design of a teaching quality analysis and management system for PE courses, with the goal of standardizing the workflow related to sports performance management, achieving scientific management and information management, transforming the traditional complex teachers' workplace, and increasing work efficiency through the application of the target system. The system can mine the correlations between PE course grades, analyse these relationships scientifically, provide good decisions for educators and teachers and teacher management, better guide teaching work, and make students' teaching quality assessment data a truly important resource.

## Figures and Tables

**Figure 1:** System function module.

**Figure 2:** Process of test type deletion programme.

**Figure 3:** Process of data mining.

**Figure 4:** Comparison of CPU and GC activities.

**Figure 5:** Running time of the system with different durations.

**Figure 6:** Quality scene of each cluster when the real data set is increasing.

**Figure 7:** Performance comparison and analysis of large-scale data set algorithms.

**Figure 8:** Comparison of clustering time between positive constraints and negative constraints.

**Table 1:** IP-specific configuration table.

Machine name	Masker	Slave 1	Slave 2	Slave 3
IP address	192.168.5.23	192.168.5.34	192.168.5.25	192.168.5.31
Attribute	Name node	Data node	Data node	Data node

**Table 2:** Data set size based on mining association rules.

Data set	*D*_1_	*D*_2_	*D*_3_
Average number of items	35	41	49
Number of data files	5	10	12
Transaction record number	6000	13000	13000

## Data Availability

The data used to support the findings of this study are available from the corresponding author upon request.
